The article "Identification and Validation of Immune Markers in Coronary Heart Disease" was retracted in 2023. Reasons: signs of a paper mill; compromised peer review; unreliable results or conclusions.

# Identification and Validation of Immune Markers in Coronary Heart Disease

**DOI:** 10.1155/2022/2877679

**Published:** 2022-08-26

**Authors:** Yuxiong Pan, Jian Zhang, Jin Li, Wei Zhao

**Affiliations:** ^1^Department of Cardiology, The Affiliated Longyan First Hospital of Fujian Medical University, Longyan, Fujian 364000, China; ^2^Division of Cardiology, The First Affiliated Hospital with Nanjing Medical University, Nanjing, China

## Abstract

**Background:**

Coronary heart disease (CHD) is an ischemic heart disease involving a variety of immune factors. This study was aimed at investigating unique immune and m6A patterns in patients with CHD by gene expression in peripheral blood mononuclear cells (PBMCs) and at identifying novel immune biomarkers.

**Methods:**

The CIBERSORT algorithm and single-sample gene set enrichment analysis (ssGSEA) were applied to assess the population of specific infiltrating immunocytes. Weighted Gene Coexpression Network Analysis (WGCNA) was utilized on immune genes matching CHD. A prediction model based on core immune genes was constructed and verified by a machine learning model. Unsupervised cluster analysis identified various immune patterns in the CHD group according to the abundance of immune cells. Methylation of N6 adenosine- (m6A-) related gene was identified from the literature, and t-distributed stochastic neighbor embedding (t-SNE) analysis was used to determine the rationality of the m6A classification. The association between m6A-related genes and various immune cells was estimated using heat maps.

**Results:**

22/28 immune-associated cells differed between the CHD and normal groups, and a significant difference was detected in the expression of 21 m6A-related genes. The proportion of immune-related cells (activated CD4+ T cells and CD8+ T cells) in the peripheral blood of the CHD group was lower than that of the normal group. The immune genes were divided into four modules, of which the turquoise modules showed a significant association with coronary heart disease. Eight hub immune genes (*PDGFRA*, *GNLY*, *OSMR*, *NUDT6*, *FGFR2*, *IL2RB*, *TPM2*, and *S100A1*) can well distinguish the CHD group from the normal group. Two different immune patterns were identified in the CHD group. Interestingly, a significant association was detected between the m6A-related genes and immune cell abundance.

**Conclusion:**

In conclusion, we identified different immune and m6A patterns in CHD. Thus, it could be speculated that the immune system plays a crucial role in CHD, and m6A is correlated with immune genes.

## 1. Introduction

Coronary heart disease (CHD), including its most serious complication, acute myocardial infarction, is a major health threat worldwide [1]. Despite significant advances in treatment, CHD remains a healthcare and financial burden [2]. Therefore, new diagnostic methods, including biomarkers, are required for targeted prevention and treatment. Atherosclerosis, the main cause of coronary heart disease, is characterized by an inflammatory process caused by cholesterol retention in the artery wall. [3]. Inflammation in arteries is mediated by innate and adaptive cells of the immune system that are recruited to the arterial lining [4]. The association between the number of circulating immune cells and the CHD phenotype has been investigated frequently in the past few years [5]. Although several studies have described the association between specific types of immune cells and CHD, we still lack comprehensive evidence. Thus, understanding the immune regulation of CHD might explicate the pathological mechanisms and identify novel immune strategies for the treatment of the disease [6].

Methylation of N6 adenosine (m6A) could occur in messenger RNAs (mRNAs), long noncoding RNAs (lncRNAs), and microRNAs (miRNAs) and is considered the common form of RNA modification [7, 8]. Regulatory proteins significantly impact m6A modification, and the exploration of these regulators could be valuable in figuring out the mechanisms of m6A [9]. Recent studies confirmed that genetic changes and dysregulated expression of m6A regulators are associated with CHD [10–12]. A comprehensive concept of the m6A regulators would further facilitate the identification of RNA methylation-based pathologic processes [13].

In this study, we systematically evaluated the proportion of immune cells and genetic changes of m6A regulators in PBMCs in patients with CHD. Next, a predictive signature with eight hub genes related to immune pathways was constructed using the Gene Expression Omnibus (GEO) database, and the stability and reliability of the model were validated through another cohort. The functional enrichment analysis was performed to reveal the potential functions of the hub gene. Further, we analyzed the association between hub gene expression and the type of immune infiltration. Moreover, we explored the correlation between immune infiltration type with m6A-related gene expression.

## 2. Methods

### 2.1. Collection and Processing of Publicly Available Data

Gene expression profile of CHD and control samples were collected retrospectively from the NCBI GEO database. We derived two GEO datasets.

The GSE9874 dataset performed the mRNA expression profile in monocyte-derived macrophages from peripheral blood of 15 CHD and 15 controls. The GSE113079 dataset performed mRNA expression profile in peripheral blood mononuclear cells (PBMCs) of 93 CHD and 48 healthy controls. The annotation platform for the GSE113079 dataset is GPL20115 while for the GSE9874 dataset is GPL96. In summary, there are two differences between two datasets: (1) The GSE9874 dataset performed the mRNA expression profile in monocyte-derived macrophages from peripheral blood while the GSE113079 dataset performed the mRNA expression profile in peripheral blood mononuclear cells (PBMCs). (2) The annotation platform for the GSE113079 dataset is GPL20115 while for the GSE9874 dataset is GPL96. The table of immune-related genes was acquired from the ImmPort database.

### 2.2. Estimation of Immune-Related Cell Infiltration through ssGSEA and Deconvolution Algorithm

ssGSEA was quoted to define the relative abundance of 28 immune-related cell types in the CHD immunological change. Panels of genes with specific characteristics used to mark each immune-related cell type were selected from a recent experiment [14, 15]. The CIBERSORT algorithm [16] was utilized to assess the abundance of 22 distinct leukocyte subsets. The Wilson test method was used to compare the difference in immune cell levels between CHD and the normal group.

### 2.3. WGCNA

The network was built by the WGCNA R package. WGCNA assessed the immune-related genes obtained from the ImmPort database. Hierarchically clustered genes are visualized in a dendrogram. A branch of the tree marked with a specific color represents a module containing highly related genes. Grey sections indicate background genes that do not belong to any module.

### 2.4. Identification of Differentially Expressed Genes (DEGs)

To screen the DEGs between the CHD and normal samples, the “limma” package in R was applied [17]. The false discovery rate (FDR) was controlled by adjusting *P* value (adj. *P* value < 0.05).

### 2.5. Quantification by the Immune Response Predictor

The ESTIMATE algorithm [18] exploits the unique properties of the transcriptional profiles to judge the tumor purity and tumor cellularity. Next, the algorithm was applied to calculate the immune scores to predict the level of infiltrating immune cells in the coronary heart and control groups.

### 2.6. Development of Machine Learning Models

In the GSE113079 dataset, 1129 immune-related genes were identified based on the ImmPort database to make WGCNA analysis. We intersected 467 immune-related genes in turquoise module associated with CHD in the GSE113079 dataset with 177 DEGs (differently expressed genes) from the GSE9874 dataset between 15 CHD samples and 15 control samples. 11 common immune-related genes were found by intersection. The importance score obtained by the random forest algorithm was applied to select the first 8 important genes (PDGFRA, GNLY, OSMR, NUDT6, FGFR2, IL2RB, TPM2, and S100A1) associated with CHD to construct the prediction model. Next, we sought to construct predictive models using the following supervised machine learning methods for categorization: logistic regression (LR), support vector machine (SVM) with the linear kernel (SVMlr) [19], SVM with radial basis function (RBF) kernel (SVMrbf), naïve Bayes (NB) [20], decision tree (DT) [21], random forest (RF) [22], gradient boosting machine (GBM) [23], K-nearest neighbor (KNN) [24], and extreme gradient boosting (XGboost) [25].

### 2.7. TF-Gene Interactions

The NetworkAnalyst platform was exploited to identify identified common gene interaction with TF-gene. The network generated for the network was acquired from the ENCODE database which is included in the NetworkAnalyst platform.

### 2.8. Identification of Immune Modification Pattern

Unsupervised clustering analysis was conducted to identify diverse immune modification methods based on the relative abundance of each immune cell type. The number of clusters and robustness was evaluated using the applied consensus clustering algorithm [26]. The R package “ConsensusClusterPlus” performed the above steps for 1000 iterations for robustness [27]. t-distributed stochastic neighbor embedding (t-SNE) was conducted to validate the immune modification method. Infiltrating immunocyte abundance score and m6A regulator expression were compared among the two distinct modification patterns by the Kruskal test.

### 2.9. Biological Enrichment Analysis for Distinct Immune Modification Methods

The Gene Ontology (GO) and Kyoto Encyclopedia of Genes and Genomes (KEGG) pathways [28] were built using the R package “clusterProfiler” [29]. Analysis of variance was set up with an adjusted *P* value < 0.01 as the cutoff criterion.

### 2.10. Identification of m6A-Mediated Genes

To screen the m6A regulator-meditated genes, 440 m6A-mediated genes were identified by whole-gene correlation analysis using the R package “Hmisc.” The criteria for distinguishing significant DEGs were set as correlation coefficient > 0.3 and the adjusted *P* value < 0.001.

### 2.11. Ethics Approval and Consent to Participate

Our study was approved by the Ethics Committee of the Affiliated Longyan First Hospital of Fujian Medical University. All participants signed an informed consent form.

### 2.12. Patient and Blood Collection

We retrospectively selected 20 patients diagnosed with CHD and 10 patients diagnosed with paroxysmal atrial fibrillation without CHD as the control group on admission, whose PBMCs were stored in the biobank. PBMCs were extracted according to the manual (FMS-FLH100100ml, Fcmacs, China) and stored in a biosafe refrigerator at 80°C. The baseline characteristics of patients are presented in Table S1.

### 2.13. RNA Extraction and Quantitative Real-Time PCR (qRT-PCR)

RNA was extracted from PBMCs by TRIzol (Invitrogen, Carlsbad, CA, USA) according to the protocols of the manufacturer. A spectrophotometer (NanoDrop-2000, Thermo Fisher Scientific) was used to inspect the quantity and quality of RNA. The steps for PCR were performed as previously described [30]. The relative expression was calculated using the following equation: relative gene expression = 2^−(ΔCtsample − ΔCtcontrol)^. All samples were measured in triplicate.

## 3. Results

### 3.1. Immune Cell Landscape of PBMC Transcriptome in Normal and CHD Groups

To assess the immune landscape and identify the immune-related genes, the GSE113079 cohort was utilized in our study, which included 93 CHD patients and 48 normal patients. Immune infiltration analysis by ssGSEA showed a higher level of activated dendritic cells, CD56 bright natural kill cells, central memory CD8+ T cells, immature B cells, mast cells, monocytes, neutrophils, regulatory T cells, T follicular helper cells, and type 17 T helper cells, as well as a lower level of activated CD4+ T cells, activated CD8+ T cells, CD56 dim natural killer cells, central memory CD4+ T cells, effector memory CD8+ T cells, immature dendritic cells, MDSC, memory B cells, natural killer T cells, plasmacytoid dendritic cells, and type 2 T helper cells in CHD compared with the control group (Figure 1(a)). Similar results were obtained by the CIBERSORT algorithm (Figure S1). Interestingly, the ESTIMATE algorithm found that the CHD group had lower immune scores than the control group (Figure 1(b)).  Figure 1(c) shows the relative proportion of immune cell abundance in each sample independently. These results indicated that the immune environment of CHD has changed greatly compared with normal people.

### 3.2. Construction of WGCNA Based on Immune-Related Genes and Identification of Key Modules

A total of 1129 immune-related genes were identified based on the ImmPort database. WGCNA analysis illustrated that these genes were included in five different modules according to correlation with CHD. The coexpression modules are shown in Figure 2(a). The interaction association was analyzed and visualized by heat map (Figure 2(b)) among the five different modules. The 467 immune-related genes in the turquoise module had a significant positive correlation with CHD, and the correlation coefficient is 0.8 (Figure 2(c)). The correlation between module membership in the turquoise module and gene significance for CHD is visualized in Figure 2(d). The pathway enrichment analysis showed that immune-related genes in the turquoise module associated with CHD are enriched in NK cell-mediated cytotoxicity, cytokine-cytokine receptor interaction, and T cell receptor signaling pathway, which indicated that these genes are widely involved in the immune process (Figure S2).

### 3.3. Construction and Validation of an Eight-Gene Signature for Distinguishing between CHD and Normal Groups

We intersected 467 immune-related genes in the turquoise module associated with CHD in the GSE9874 dataset with DEGs (differently expressed genes) from the GSE113079 dataset between 15 CHD samples and 15 control samples. 11 common immune-related genes were found by intersection. A strong relationship between 11 immune-related genes is shown in Figure 3(a). The importance score obtained by the random forest algorithm (Figure 3(b)) was applied to select the first 8 important genes (*PDGFRA*, *GNLY*, *OSMR*, *NUDT6*, *FGFR2*, *IL2RB*, *TPM2*, and *S100A1*) associated with CHD to construct the prediction model. Also, nine machine learning algorithms were applied to construct the prediction model to distinguish the CHD group from the control group. The GBM model achieved the maximum AUC value of 0.961 in the development cohort, and the NB model achieved the maximum AUC value of 0.964 in the validation cohort (Figures 3(c) and 3(d)), which showed that the eight immune-related genes can well distinguish CHD patients from the control group. Clinical samples were used for qPCR experimental verification, and the results showed that PDGFRA, IL2RB, FGFR2, and S100A1 were differentially expressed in CHD (Figure 3(e)). These four candidates are also expected to be biomarkers for the identification of CHD. The full names of the genes mentioned above are listed in Table S2.

### 3.4. Functional Analysis of Immune-Related Core Genes

To further explore the correlation between the immune-related core genes and immune cells, a correlation heat map is established in Figure 4(a). A significant positive correlation was shown between GNLY, IL2RB, and activated CD8+ T cells (Figures 4(b) and 4(c)). A significant negative correlation was established between NUDT6 and activated CD8+ T cell or FGFR2 and activated CD8+ T cell (Figures 4(d) and 4(e)). These results demonstrated that these core immune genes are strongly associated with immune cells significantly changed between coronary heart disease and the control group. The ChIP-X Enrichment Analysis (CHEA3) platform was used to predict the transcription factors regulating the differential immune genes. The top five transcription factors associated with these immune-related genes were PRRX1, ZNF469, TWIST2, OSR1, and MKX (Figure S3). TF-gene interactions and the TF-miRNA coregulatory network were collected using “NetworkAnalyst” for the eight core genes (PDGFRA, GNLY, OSMR, NUDT6, FGFR2, IL2RB, TPM2, and S100A1). MYC, TP63, SOX2, RNF2, MTF2, and SUZ12 were the top six transcription factors by the TF-gene network while hsa-miR-218 and hsa-miR-33 were the top two microRNAs that may regulate the expression of core immune-related genes.

### 3.5. Identification of Two Different Immune Types in the CHD Group

To discover the heterogeneity of immune status among patients with CHD, we did cluster analysis based on the immune infiltration abundance score in CHD by ssGSEA. Cluster analysis identified two different immune patterns in the CHD group (Figure 5(a)). We name two different immune patterns as “CHD Type1” and “CHD Type2”.

“CHD Type1” contained 31 CHD patients while “CHD Type2” contained 62 CHD patients. This classification is considered reasonable by the t-SNE method (Figure 5(b)). ssGSEA showed significant differences between CHD Type1 and CHD Type2 in activated CD8+ T cells, central memory CD8+ T cells, effector memory CD8+ T cells, immature dendritic cells, and macrophages calculated by ssGSEA (Figure 6(a)). GSEA KEGG analysis showed that DEGs between two CHD types were enriched in antigen processing and presentation, NK cell-mediated cytotoxicity, primary immunodeficiency, T cell receptor signaling pathway, and Th1 and Th2 cell differentiation (Figure 5(c)). GSEA GO analysis showed that the DEGs above were enriched in negative regulation of chromosome organization, protein-DNA complex assembly, protein-DNA complex subunit organization, and T cell receptor signaling pathway (Figure 5(d)).

### 3.6. Landscape of Gene Expression of m6A Regulators and Correlation between m6A Regulator Gene Expression and Immune Cell Abundance

RNA methylation is a novel epigenetic modification involved in the regulation of various biological processes such as stem cell renewal, immunity, tumorigenesis, metastasis, and cell development and differentiation [31–33]. Although there are some research studying the relationship between RNA methylation and immune infiltration in heart disease [34–36], a few studies were focused on the PBMC transcriptome between CHD patients and controls. We investigated the roles of 21 m6A RNA methylation regulatory genes in CHD. Protein interaction of the 21 m6A-related genes was shown (Figure 6(b)). t-SNE analysis demonstrated that methylation-related genes could distinguish between the normal and CHD groups (Figure 6). Subsequently, we conducted a genome-wide association analysis and screened 440 m6A-related genes (Cor > 0.3 and *P* < 0.001). Functional enrichment analysis suggested that m6A-related genes were enriched in cytokine-cytokine receptor interaction, GPCR ligand binding, inflammatory response, chemotaxis, and P13K-Akt signaling pathway (Figure 7(a)). Then, we analyzed the association between 21 m6A regulators and 28 immune cell types. METTL14 was significantly positively correlated with activated CD8+ T cells, while WTAP was significantly positively correlated with activated CD4+ T cells (Figure 7(b)). These results demonstrated that m6A are strongly associated with immune genes and immune cell infiltration between the coronary heart disease and control groups.

## 4. Discussion

CHD is a chronic inflammatory disease with various immune-related changes [37]. However, the differences in the immune cell subsets in the peripheral blood of the CHD and normal groups are yet to be evaluated. Several studies have explored m6A in tumor-specific microenvironment-infiltrating cells [38, 39]. Thus, we speculated that similar results were observed concerning m6A modification in participating in the immune microenvironment in CHD. Herein, we discussed the immune modification methods in PBMCs from the CHD group. To uncover how m6A effectuates the immunology change in CHD and enriches infiltrating immunocytes, m6A-related gene GO analysis was performed. We found that the expression of the majority of infiltrating immunocytes altered between healthy and CHD samples; these infiltrating immunocytes participate in CHD development. A classifier built by immune-related genes could distinguish between healthy and CHD samples, verifying the role of immune genes in CHD. Among the 467 immune-related genes, *PDGFRA*, *GNLY*, *OSMR*, *NUDT6*, *FGFR2*, *IL2RB*, *TPM2*, and *S100A1* may be crucial because of the fold-change and significance in the two cohorts. Furthermore, the correlations between immune characteristics and m6A regulators of the CHD were investigated with respect to infiltrating immunocytes and immune-related pathways. We found that various m6A regulators were closely associated with these immune signatures. METTL14 had the same trend as activated CD8+ T cells, while WTAP was consistent with changes in activated CD4+ T cells. The activated CD8+ T and CD4+ T cells are a major component of adaptive immunity and play a key role in CHD homeostasis. The two distinct immune patterns in the CHD group deemed that the PBMC samples could be utilized for alternative pathobiology-based classification of CHD. Finally, the genes associated with immune modification patterns were identified. The regulation of the expression of these genes was influenced by the immune phenotype. The abundant results in the current study showed similar correlations that would provide directions to other investigators to identify the key m6A regulator and immune features related to CHD.

This is a novel study to explore the correlation between m6A regulators and immune response. Numerous results open new directions for the pathogenesis of immune-related CHD based on m6A modification mechanisms. The present study also introduced the novel m6A mechanism underlying CHD immune microenvironment regulation. Currently, epigenetics research regarding CHD has a marked knowledge gap. Thus, comprehensive consideration of the novel m6A mechanism and immune microenvironment theory to reveal the pathogenic mechanisms underlying CHD would be a breakthrough.

Nevertheless, the present study also has some limitations. First, since this study was aided by bioinformatics analysis, we only selected three datasets for analysis, which resulted in less rigorous analysis results. We will include more datasets in subsequent studies and pay attention to the batch effect. Meanwhile, the sample sources of these two datasets are not completely consistent, one of which is PBMCs, and the other is monocyte-derived macrophages. However, according to the results of bioinformatics analysis of numerous tumor studies based on The Cancer Genome Atlas (TCGA), data analysis could be deemed reliable. Nonetheless, the current findings need to be substantiated by subsequent experiments. Moreover, some data, such as the clinical characteristics of CHD, were unavailable, making it difficult to uncover the role of m6A in immune regulation from multiple aspects. Therefore, biochemical experiments should be performed to explore changes in m6A. Taken together, our findings confirmed the strong influence of m6A modification on the immune characteristics of CHD, which has provided a completely new direction for the underlying pathogenesis.

## 5. Conclusion

In conclusion, we found different immune and m6A patterns between the normal and CHD groups and experimentally confirmed differentially expressed immune-related genes in CHD. Our study provides new ideas for better clinical research and treatment of CHD.

## Figures and Tables

**Figure 1:** (a) The differences in immune cell abundance between the coronary heart disease and control group were calculated by the ssGSEA method based on the transcriptome profile. The Wilson test method was used to compare the difference in immune cell levels between CHD and the normal group. (b) By using the ESTIMATE algorithm, the CHD group had lower immune scores than the normal group. (c) The proportion of immune cells was calculated by the ssGSEA algorithm for all samples. The first 93 samples were from patients with coronary heart disease, and the last 43 samples were from the normal group.

**Figure 2:** (a) The cluster dendrogram of genes in GSE113079. Each branch in the figure represents one gene, and every color below represents one coexpression module. (b) Heat map plot of the adjacencies in the hub gene network. (c) Heat map of the association between modules and the illness status of CHD. The turquoise module was shown to be more correlated with CHD. (d) By the WGCNA method, we calculated the module membership and gene significance score of each gene. This figure shows a relationship between module membership score in the turquoise module and gene significance score for CHD.

**Figure 3:** (a) Correlation heat map of common DEGs in GSE9874 and GSE113079. (b) The importance score for 11 common immune-related genes associated with CHD was obtained by random forest algorithm. (c) and (d) show construction and validation of the prediction model for CHD by nine machine learning algorithms independently. (e) qRT-PCR analysis of DEGs between the control and CHD groups. Data are presented as mean ± SEM. Statistical analysis was performed with one-way ANOVA followed by Bonferroni's correction. ^∗^*P* < 0.05, ^∗∗∗∗^*P* < 0.0001.

**Figure 4:** (a) Correlation heat map between the 8 immune-related core genes and immune cells. (b) A significant positive correlation between GNLY and activated CD8+ T cells. (c) A significant positive correlation between IL2RB and activated CD8+ T cells. (d) A significant negative correlation between NUDT6 and activated CD8+ T cells. (e) A significant negative correlation between FGFR2 and activated CD8+ T cells.

**Figure 5:** (a) TF-gene interactions were collected using NetworkAnalyst for the common DEGs (PDGFRA, GNLY, OSMR, NUDT6, FGFR2, IL2RB, TPM2, and S100A1). (b) TF-miRNA coregulatory network for the common DEGs (PDGFRA, GNLY, OSMR, NUDT6, FGFR2, IL2RB, TPM2, and S100A1).

**Figure 6:** (a) By using cluster analysis, two different immune patterns were identified in the CHD group. We name two different immune patterns, “CHD Type1” and “CHD Type2”. (b) T-SNE was used to confirm the rationality of classification for two different immune patterns in CHD. (c) GSEA KEGG analysis of differential expressed genes between the CHD Type1 and the CHD Type2 group. (d) GSEA KEGG analysis of differential expressed genes between the CHD Type1 and the CHD Type2 group.

**Figure 7:** (a) By using the ssGSEA algorithm, it showed significant differences in immune cell abundance between CHD Type1 and CHD Type2. (b) Protein interaction of the 21 m6A-related genes. (c) Significant differences are identified in m6A-related genes between CHD and the normal group. (d) By t-SNE analysis, methylation-related genes could distinguish between the normal group and the CHD group.

## Data Availability

The data that support the finding of this study are available from the corresponding author upon reasonable request.

## Supplementary Materials

Supplementary Materials Figure S1: abundance of 22 immune cells is calculated by the CIBERSORT algorithm in the GSE113079 cohort. FigureS2: GO analysis of the turquoise module genes by WGCNA. FigureS3: top ten transcription factors predicted by the ChIP-X Enrichment Analysis (ChEA3) website. Table S1: the baseline characteristics of patients. Table S2: the full names of the core genes.
